# Study on Tourism Consumer Behavior and Countermeasures Based on Big Data

**DOI:** 10.1155/2022/6120511

**Published:** 2022-07-19

**Authors:** Jing Li, Bin Cao

**Affiliations:** ^1^Jinzhong University, Jinzhong 030619, Shanxi, China; ^2^Universiti Sains Malaysia, Gelugor 11800, Penang, Malaysia

## Abstract

In our study, through consulting, summarizing, and analyzing a large number of related literature studies on tourism consumer behavior, tourism big data, text data analysis, and so on, a framework of research ideas on tourism consumption was constructed. The train browser, NLPIR, and other software packages are used to crawl, preprocess, and mine the travel sample data, and the word frequency analysis, co-occurrence analysis, content analysis, sentiment analysis, network analysis, and other methods are used to analyze the characteristics and decision-making behavior of tourists. Based on the results of behavioral analysis, we proposed tourism development strategies from three aspects: reforming and promoting tourism marketing strategies, improving tourism product and service quality, and improving tourism destination management methods. The results show that (1) for the tourist characteristics, taking into account the factors of climate and geographical location, the domestic market is divided into four grades of markets, and different marketing strategies are adopted according to different market characteristics; (2) for the tourism decision-making behavior, a “push-pull resistance” tourism decision-making model was established through word frequency analysis, co-occurrence analysis, and content analysis; (3) for the tourism consumption preferences, through network analysis of scenic spots, it is found that there are three tourist routes preferred by tourists; and (4) for the tourism perception evaluation behavior, based on the “cognitive-emotional” model, this study describes the tourism image from the two dimensions of the cognitive image and emotional image. Generally speaking, tourists show a positive perception state. The research on tourism consumer behavior based on UGC (user-generated content) data can help scenic spots and other tourism companies to understand the characteristics and rules of tourists' behavior, understand the consumption preferences of different tourism groups, develop diversified tourism products, improve the quality of tourism services, and further cater to market segments. This research provides a new idea for tourist attractions and tourism management departments to monitor tourist behavior through big data analysis.

## 1. Introduction

Tourism consumer behavior involves many disciplines such as marketing [1]. Tourism consumption behavior refers to the process that tourism consumers choose and purchase tourism products to meet the needs of tourism pleasure and other experiences. This process includes the generation of needs before travel, the decision-making process, consumption in scenic spots, and post-purchase evaluation. Influenced by many factors such as economy, society, and cultural environment, it is an experience activity with comprehensive, marginal, and extraordinary characteristics [2].

The American Marketing Association defines consumer behavior as follows: “The dynamic interaction process among emotional, cognitive, behavioral, and environmental factors is the behavioral basis for human beings to perform the exchange function in life” [3]. This definition regards consumer behavior as a process, including multiple stages of selection, purchase, and disposal, and the process is dynamic. Tourism consumption behavior is more complex because it involves the whole process from leaving home to returning home [4]. To reveal the rules of tourist behavior, the relationship between various behaviors, and the core influencing factors of behavior, academia has proposed many different models. Despite the differences among different models, these models collectively emphasized these psychological activities and behavioral manifestations, such as travel motivation, travel decision-making, choice preference, destination image, and satisfaction, before, during, and after travel [5].

Tourism motivation is an internal factor that prompts potential tourists to take a certain tourism action, and it is also a key factor for a series of tourism behaviors in the future. Unlike consumption demand, consumption motivation is related to products, so tourism motivation is the link between tourism demand and specific tourism destinations [6]. Scholars at home and abroad have made a lot of research on tourism motivation. The most popular theoretical models are the distribution center model, push-pull theory, optimal arousal theory, leisure incentive method, and travel career ladder (TCL) model, among which push-pull theory is the most widely used [7].

Based on scholars' cognition that “tourism behavior is a series of rational decision-making activities,” most of the tourism decision-making theories have evolved from the decision-making model of consumer behavior, which has led to the emergence of many tourism decision-making behavior models [8]. Sirakaya and Woodside, Smallman, Cohen, and other scholars have made a more detailed summary of the tourism decision-making model, mainly focusing on the model research of destination selection and various subdecisions (such as accommodation and tourism activities) [9]. Summarizing previous research on decision-making models, Sirakayaet al. believe that the final tourism consumption decision will depend on the interaction between the following variables: intrinsic variables, including travel attitude, motivation, information search behavior, and personality characteristics; extrinsic variables, including constraints, destination pull factors, the influence of family and reference groups, marketing mix, social class, and culture; the nature of the scheduled trip, including travel distance and date and playtime; and travel experience, including emotions and feelings during the trip and post-tour evaluation [10].

Motivation initiates action and guides desirable behavior, but policymaker preferences help filter choices precisely; preferences are more specific than motivation, revealed by visitor whereabouts and visitor behavior. Many scholars' research on tourism consumption preference focuses on destination choice preference (such as Tzu-Kuang Hsu), shopping preference (such as Samuel), accommodation preference (such as Isabel), food preference (such as Richard), etc. Destination image is “an attitude or psychological structure that reflects the sum total of tourists' personal views, trust and impressions of a tourist destination” [11]. During the entire tourism process, tourists' perception of the destination image is dynamic. Destination image theory is an important part of tourism research and is widely regarded as an important factor affecting tourists' decision-making, destination selection, post-tour evaluation, and future behavior [12]. The advent of the Travel 2.0 era (i.e., new ways for real travelers to interact and share information or content through Web 2.0) has changed the way travel information is searched, viewed, and evaluated. In this context, the tourism destination image has been reshaped and widely disseminated through Web 2.0 and UGC [13]. In the study of destination image perception, the most widely used theoretical model is the “cognitive-affective” model; that is, the destination image is divided into two interrelated components: cognitive image and affective image, where the cognitive image is an individual knowledge or belief about a destination. Emotional image refers to an individual's subjective feelings about the destination. The interaction of cognition and emotion forms a unique overall image of each destination, including positive or negative evaluations. Compared with emotional image, cognitive image has a stronger impact on the overall image [14].

At present, scholars at home and abroad have not reached a clear consensus on consumer satisfaction. Some scholars (such as Oliver) believe that satisfaction is an emotional state derived from tourism experience [15]. In this view, tourists' emotion has become an important indicator of satisfaction evaluation. Some scholars (such as Chon) believe that satisfaction is a function of goodness of fit between tourists' expectations of the destination before travel and the perceived evaluation of their visit experience after travel, and the expectation uncertainty model is the most commonly used measurement model.

With the rapid development of the Internet, structured and unstructured data are generated, recorded, stored, and accumulated, forming big data with the characteristics of volume, variety, and velocity, bringing amazing changes to tourism research, which has entered the big data era [16]. According to different data sources, tourism big data are mainly divided into three categories: UGC data, equipment data, and transaction data. Among the three types of data, UGC data have the most applications due to its low cost and easy access [17]. Device data applications have problems such as high cost, low accuracy, and small coverage. Since most of the transaction data are private information, only tourism organizations or government departments are used. Owned, its use level is the lowest.

In the digital age, the proliferation of the Internet and social media has dramatically changed travel patterns, providing a platform to share UGC data. User-generated content (UGC), also known as user-generated content (UCC) and consumption-generated media (CGM), was first proposed by KPCB chief analyst Mary Meeker in 2005, thinking that UGC is a new type of content in the Web 2.0 environment. There is no unified and clear definition of the creation, release, and organization mode of information resources. UGC data have been widely used in tourism research and mainly include two types: (1) online text data, such as online reviews, online travel notes, and blogs posted on social media; (2) online photo data, such as in photo sharing online photo data published by websites or online travel journals. However, due to various limitations, UGC data such as audio and video have not been widely used by researchers at home and abroad. The UGC data discussed in this study are mainly text data [18]. Online text data mainly include two types: one is review data, that is, the evaluation data of online tourism products or tourism destinations, expressing tourists' attitudes towards tourism products (such as accommodation facilities, restaurants, and scenic spots), mainly used to measure satisfaction, electronic word of mouth, etc. [19]. The second is online travel notes or blogs, that is, travel note modules on online travel websites or travel blogs on social media, which record travel feelings and experiences, mainly involving travel behavior, travel sentiment analysis, and travel recommendations. Research on UGC tourism data, at both home and abroad, focuses on empirical research, but the research focus is slightly different. Foreign research focuses on tourist satisfaction/service quality, destination image, tourism behavior, and tourist segmentation. In China, the purpose of land image and tourism behavior is the focus of research [20].

Co-occurrence refers to the phenomenon that specific keywords co-occur in a text collection. Co-occurrence analysis is a quantitative study of co-occurrence phenomena to reveal the content correlation of information and the knowledge implied by feature items [21]. The specific process of co-word analysis mainly has four stages: one is to determine the analysis data set; the other is to determine the analysis object. High-frequency words related to the research object are extracted from the text collection; the third is to construct a binary co-word matrix to obtain quantitative information such as co-occurrence frequency; the fourth is to conduct co-word analysis, which is generally combined with social network analysis for visual display [22].

Throughout the research on tourism consumer behavior at home and abroad, it is more inclined to conduct research on tourists' tourism motivation, tourism decision-making, spatial behavior, consumption preference, tourism experience, destination image, tourist satisfaction, and other subfields from an individual and micro-perspective [20]. However, they all ignore a problem: tourists are an organic whole, and their behavior runs through the entire tourism process before, during, and after tourism, but the relevant research literature seldom regards pre-tourism, tourism, and post-tourism as the study as a whole. Previous studies usually divide tourism consumer behavior into multiple subfields and use questionnaire surveys and other survey methods to conduct in-depth, detailed, and enlarged research on a subfield, but it is easily affected by questionnaire design structure, sample sampling, and investigators. Due to the limiting factors such as the subjectivity of the survey, it is impossible to objectively and completely understand the behavioral characteristics and laws of tourists. However, with the widespread of social media and Web 2.0, an online search for travel information, purchase and evaluation of travel products, and sharing travel experiences have become one of the important behavioral characteristics of tourists. UGC data with other characteristics have also become one of the important data sources for tourism behavior research [23]. In addition, in the research on tourism consumption behavior based on UGC data, domestic and foreign researchers have focused on empirical research on tourist satisfaction, destination image, tourism spatial behavior, tourism decision-making, etc., lacking the overall research on tourist behavior [24].

Therefore, this study combines the characteristics and content of online travel data to conduct an overall analysis of tourist behavior from the aspects of tourism motivation, tourism decision-making, consumption preference, destination image perception, and tourist satisfaction. This research proposes a research framework of tourism consumption behavior based on online travel notes, which is mainly divided into two levels: the first level is a three-stage dynamic model of tourism consumption behavior; the second level is to establish tourism decision-making, tourism consumption preference, and behavioral models such as perceptual evaluation after swimming.

In our study, we first conducted the data collection and mining and introduced the general situation of the tourist area and introduced the data collection and preprocessing of online travel notes, the selection basis of text mining tools, and the selection criteria of online travel note samples in Section 2 and then introduced the methods of word frequency analysis, co-occurrence analysis, network analysis, sentiment analysis, etc., and conducted mining and research on the characteristics of tourist consumption behavior from four aspects: tourist characteristics, decision-making behavior, consumption choice preference, and perception evaluation, which can be found in Section 2; in Section 3, through in-depth research on the behavior characteristics extracted by text data mining, the influencing factors of tourism consumption behavior are summarized, and combined with the results of field research, the corresponding strategies for tourism development planning in tourist areas are put forward.

## 2. Methods and Data Collection

### 2.1. Methods

#### 2.1.1. Literature Research

The literature research method is a basic research method adopted in this article. A large number of related disciplines and professional books and relevant predecessors' research results have been consulted. On the basis of sorting out and summarizing previous research, the research direction and content of this study are determined; at this stage, by consulting a large number of related literature on summer tourism, consumer behavior, tourism big data, etc., the theoretical basis and methods of this research are summarized [3].

#### 2.1.2. Content Analysis

Content analysis is a method that quantitatively analyzes the content of nonquantitative literature to find out the core content and laws contained in the literature. This research uses NLPIR big data semantic intelligent analysis software to analyze the content of the collected online travel text data and obtained valuable and meaningful data, then explores the behavioral characteristics and laws of summer tourism consumers, and finally explains the research phenomenon.

#### 2.1.3. Sentiment Analysis

Text sentiment analysis refers to the process of analyzing, processing, summarizing, and reasoning on subjective texts with emotional color [20]. According to the different granularity of text, it can be divided into multiple levels such as word level, sentence level, and chapter level. This study uses sentiment analysis to extract emotional words or emotional information from the online travel text data set and uses the chapter as a unit to identify the emotional color of travel notes, so as to obtain tourists' emotional tendencies towards four places in southern Xinjiang.

#### 2.1.4. Network Analysis [12]

Network analysis is a method to study the characteristics of the entire network and the individuals in the location-based network structure by describing the relationship structure between given entities (represented by nodes) and applying quantitative techniques to generate relevant indicators or results [15]. Based on the idea that the relationship between tourist attractions is not isolated but related to each other, this study analyzes the network structure between tourist attractions by calculating the co-occurrence frequency of different tourist attractions and proposes a proposal for tourism attraction cooperation strategy based on summarizing the spatial flow characteristics of tourists between tourist attractions.

#### 2.1.5. Mathematical Statistical Analysis [5]

This study uses SPSS and Excel software to carry out statistical analysis on the crawled tourist sources, days of play, travel companions, and other indicators, as well as the number of articles and frequency of use of related subject words, to obtain the basic characteristics of tourists, and to study summer tourism consumption. Behavioral characteristics provide corresponding data support [25].

This study mainly uses NLPIR (natural language process and information retrieval) software to achieve co-occurrence analysis. The calculated quantitative information includes co-occurrence frequency, binary probability, and binary word pair information entropy. Co-occurrence frequency refers to the number of co-occurrences of two words before and after, which is used to reflect the strength of association between them. It is generally believed that the higher the co-occurrence frequency of a phrase, the closer the relationship between the phrases. Binary probability refers to the probability of occurrence of co-occurring word pairs, and the information entropy of a binary word pair represents the breadth of information contained in the phrase [6]. The calculation formula of the information entropy is as follows:

(1) $$\begin{array}{c} H\left(U\right)=-\sum_{i}^{n}P_{i}\log\left(P_{i}\right), \end{array}$$

where *H* (*U*) is information entropy and *P*_*i*_ is the probability of variable *i*.

To extract and utilize useful information hidden in online text data, methods such as text mining and content analysis are widely used in tourism research. Text mining mainly includes three typical stages: data collection, data mining, and result output, in which the data mining stage includes two sub-steps of data preprocessing and pattern discovery. The first step of data collection is as follows. There are two main ways to collect UGC data: open API access and Web crawler. The second step is data mining. Collected online text data are analyzed to extract useful information through two substages: data preprocessing and pattern discovery. Pattern discovery is another key stage of text mining, aiming to explore interesting information in documents, and typical techniques in existing tourism research are LDA analysis, sentiment analysis, statistical analysis, clustering and classification, text summarization, and dependency modeling. The third step results in output [8]. Interesting information extracted through data mining is transformed into useful knowledge to further serve tourism research. According to relevant research, valuable knowledge covers tourist satisfaction, consumption preference, tourist destination image, tourist route, review characteristics, etc., which is of great help in improving tourism management and providing tourism advice [19].

### 2.2. Data Collection

The four prefectures in southern Xinjiang include Aksu Region, Kizilsu Kirgiz Autonomous Prefecture, Kashgar Region, and Hotan Region. It is an important section of the central route of the Silk Road, the southern route, and the church. The two routes of the Silk Road pass through the four prefectures in southern Xinjiang. It is located on the northwestern border of the motherland, the western edge of the Taklimakan Desert, and the southwestern part of the autonomous region; it borders six countries including Kyrgyzstan and India. There are 5A and 4A tourist attractions such as the ancient city of Kashgar, the Populus euphratica scenic spot in Zepu County, the Stone City scenic spot, and the Daolang portrait scenic spot, the Honghai Bay scenic spot, and the Etigar Mosque. It is a first-class port in 5 countries including Kashgar International Airlines and has a rich border and ethnic characteristic tourism resources.

#### 2.2.1. Sample Selection of Online Travel Data

This research mainly uses the travel notes related to the actual tour itinerary shared by tourists on the Internet after the trip. By searching for websites with tourism community functions (based on the comprehensive ranking of tourism websites on top.chinaz.com), and according to the research object and research purpose of this study, Ctrip, Mafengwo, Baidu Travel, and Qunar were selected as the main data sources. In the crawling of online travel note text data, the Web crawler software (Train Browser 8.2 version) was mainly used to crawl the online travel note data related to summer travel in southern Xinjiang from four selected online travel websites, and the original online travel note database was formed, namely Database.mdb. Then, the crawled travel database according to the following criteria is filtered: online travel notes that do not take southern Xinjiang as a tourist destination are excluded; travel notes that only have pictures, less text (less than 500 words), incomplete travel information, and are not suitable for text content analysis are eliminated; travel notes that are not for the purpose of sharing travel experiences are eliminated, such as advertisements and propaganda; and duplicate travel notes and merge serial travel notes of the same author are removed. After screening, 500 online travel notes (including 250 on Mafengwo, 110 on Qunar, 90 on Baidu Travel, and 40 on Ctrip) were selected as the initial text database for this study.

Due to the limitation of HTML structure, some indicator data need to be further sorted out. For example, Excel's “replace” function is used to clean up redundant text information such as “departure time/” in indicators such as “departure date”; blank data are filled according to the content of travel notes; the CLEAN function is used to remove characters such as “newline” and “space” in the text of the travel note; and individual vacancies are manually extracted from the text to supplement and improve them. In addition, the body text data of the 500 travel notes are copied into an “original corpus.txt” document to form a travel note one-line format.

#### 2.2.2. Selection of Chinese Text Mining Tools

In this study, the NLPIR big data semantic intelligent analysis platform developed by Zhang Huaping was selected for text mining analysis. The NLPIR analysis platform has the following advantages: (1) the word segmentation tagging technology based on the cascading hidden horse model has a word segmentation accuracy of close to 98.23% and has the advantages of high accuracy, and fast speed, and strong adaptability. (2) The entity extraction system based on role annotation can intelligently identify the names of people, places, institutions, media, authors, and the subject keywords of articles that appear in the text. (3) The word frequency statistics function based on the patented perfect double array TRIE tree algorithm has high efficiency and is more than ten times faster than the conventional algorithm. (4) The keyword extraction technology based on context conditional entropy can extract several words or phrases representing the semantic content of the article on the basis of comprehensively grasping the central idea of the article. In addition, it uses cross-information entropy to calculate the context of each candidate word. Conditional entropy identifies the most recent new words and assigns them weights. (5) Text sentiment analysis is based on a deep neural network, and NLPIR sentiment analysis provides two modes: sentiment discrimination of full text and sentiment discrimination of specified objects [26, 27].

#### 2.2.3. Preprocessing of Travel Note Text Data Set

In this study, the travel note text data are preprocessed as follows: (1) new words are discovered and user dictionaries are built. Using the new word discovery function of NLPIR, words with new connotations and new concepts are mined from the original corpus and added to the user dictionary to improve the accuracy of the word segmentation system. In addition, the user dictionary is manually checked to fill in the gaps, and the content of the scenic spots and tour routes in the research area in the user dictionary is further improved; (2) building stop word lists for data cleaning: data cleaning is used to detect and remove inaccurate or useless records in text data, such as misspellings and stop words, to leave valuable travel information; and (3) word segmentation and word frequency statistics are circularly performed, and the user dictionary is continuously improved, and word list is stopped until accurate word segmentation and word frequency statistics are achieved. Finally, the more accurate word segmentation results are analyzed by Chinese word frequency statistics, and the phrases that are irrelevant or meaningless to the research content are eliminated.

## 3. Results and Discussion

### 3.1. Analysis of the Basic Characteristics of Tourists

For the consideration of personal privacy protection, online travel notes rarely show the demographic characteristics of tourists but can capture module information such as tourist source, travel time, travel days, travel partners, and travel methods and obtain basic characteristics of tourists through descriptive statistical analysis [20].

Distribution characteristics of customer sources: the distribution of source areas shows obvious geographical differences between east-west and north-south. North China, Northeast China, and East China accounted for 82.6% of the tourists [21-23]. Affected by the principle of travel distance attenuation and the difference in summer climate, Northeast China accounted for the largest proportion, followed by North China and East China. There are many high-temperature weather in summer and economic development factors, and there is a strong demand for going north to escape the summer heat. The tourism resources in the southwest and northwest regions are relatively concentrated, which can meet the tourism needs of tourists in the local and surrounding areas, so there is a big difference between the east and west source of tourists and affected by the travel distance, and southern Xinjiang is more attractive to northern tourists than southern tourists. Therefore, there are differences in the distribution of tourists from north to south. However, due to the law of regional differentiation, there are differences in tourism resources between the north and the south. For the motivation of seeking innovation, the central and southern regions and the southwest regions will become potential tourist sources (Table 1).

Figure 1 shows the results of statistics of departure date data in 500 travel notes based on the year. The number of travel notes generally maintains a continuous upward trend, with a larger increase after 2015, which is not only closely related to the tourism development of the four southern Xinjiang regions but also related to the popularity of online travel notes. With the gradual improvement of tourism-sharing community-related websites, the creation of online travel journals has gradually become a part of the tourism process.

Regarding the number of days to visit (Figure 2), due to the abundant resources of scenic spots in southern Xinjiang (three tour routes have been developed), the tickets are valid for three days, and the summer vacation is long, so more tourists choose the itinerary within 1 week, accounting for 84%, of which 3-4 days of in-depth tours are the most popular, followed by 1-2 weeks of itineraries, accounting for 13.3%, and the least number of tourists who choose to play for more than 2 weeks. After calculation, the average playing days of the travel note sample is 5 days, which shows that tourists in southern Xinjiang spend a long time playing.

The per capita consumption of tourists has a relatively large span, with a minimum per capita consumption of 200 yuan and a maximum of 10,000 yuan, but in general, the per capita consumption is concentrated in the range of 1,000–3,999 yuan (57.4%). According to the content of the travel notes, the reasons for the low consumption are as follows: first, the distance to the destination and the number of days of play are few, so the consumption is not high; second, there are friends or relatives in the local area; it is to choose low-cost group tours. Combined with the number of days of tourist travel, it is calculated that the per capita daily consumption is between 100 and 2550 yuan (see Figure 3).

### 3.2. Analysis of Tourists' Decision-Making Behavior

Travel motivation is a key factor in all travel behaviors and an important driver of travel decisions [24-25]. 59 related entries were extracted through word frequency analysis articles, and entries were classified into three types of factors: push force, pull force, and resistance force according to the word meaning (see Table 2).

Iso-Ahola divides push factors into two dimensions: escape (such as escape from everyday life or interpersonal circumstances) and seeking (such as adventure or friendship building), which explain why tourists travel and what type of destination or type of destination they need. Drawing on Iso-Ahola's division of dimensions, after content analysis, this study divides the thrust factors into two dimensions: escape and seek [26]. Through the co-occurrence analysis, tourists are not only eager to escape the high temperature in summer but also want to escape the hustle and bustle of the city, and they want to go on a trip. Seeking: through the cluster analysis of the words of seeking dimension, tourists' travel motives are mainly to accompany family members or friends, to seek novelty, to go on vacation, to pursue freedom and excitement, etc. Among them, accompanying family members and friends to experience different sceneries and perceive different worlds is an important factor driving tourists to travel abroad. Summer tourism is not only a leisure and vacation way for people to escape from high-temperature cities but also an important way for people to seek companionship and novelty.

Tourism decision-making is the external manifestation of tourism motivation and the core behavior in the process of tourism [27]. A decision-making process contains multiple subdecisions of information, and each subdecision exists in two stages of the tourism process: one is information search and decision-making before travel, such as which information acquisition channel to choose and what information to search for; the second is tourism instant decisions. According to the content analysis and word frequency analysis of travel notes, this section mainly analyzes the characteristics of tourism decision-making behavior from three aspects: tourism decision-making behavior, decision-making information needs, and information acquisition channels.

After keyword analysis and co-occurrence analysis (see Table 3), tourism information channels mainly come from the Internet, including travel notes, strategies, and reviews of travel websites such as Ctrip, official websites, or APPs of scenic spots and search engines such as Baidu, Taobao, and Dianping. Due to third-party platforms information needs, tourists have different preferences in choosing information channels. For example, tourists mainly obtain information on destinations and attractions, tourist routes, itineraries, and other information through the strategies, travel notes, and reviews of tourism community websites; book and buy tickets through the official website or APP of the scenic spot, online travel website, Taobao, etc.; through the official website of the scenic spot or Ctrip, etc.; booking accommodation on travel websites; and inquiring about recommended food through Dianping and other platforms.

### 3.3. Analysis of Tourists' Consumption Preference

Online travel notes are travel experiences and experiences recorded by tourists after their trips based on their memories. The sights and travel activities frequently mentioned by tourists in travel notes indicate that they have left a deep impression on tourists or unforgettable travel experiences. Such experiences are often positive. Therefore, the greater the frequency of tourist attractions or tourist activities, the higher the popularity of the tourist attractions or tourist activities, and the more tourists prefer them. Based on this, this study filters out the tourist attractions that tourists prefer based on the word frequency of the names of the attractions, as shown in Figure 4.

The preference of tourist attractions based on word frequency screening shows a typical long-tailed curve distribution from high to low. The trend of the curve changes can reflect the uniformity of the heat distribution of tourist attractions. The faster the curve changes and the greater the amplitude, the more uneven the heat distribution of tourist attractions and vice versa. It can be seen from Figure 4 that only a few high-fat spots are distributed in the head of the curve, and most of the low-fat spots are distributed in the long tail of the curve, of which Kashgar Old Town has the highest weight.

### 3.4. An Analysis of Tourists' Perception and Evaluation Behavior

Tourism image refers to an individual's overall perception or overall impression of a tourist destination, which not only affects the destination selection stage but also affects the behavior of tourists, including sharing behavior, revisit intention, and recommendation behavior. It is widely accepted that the image of a tourist destination is generalized into two interrelated dimensions: the cognitive dimension and the emotional dimension, of which the cognitive dimension is the premise of the emotional dimension, both of which have a direct impact on the overall image of the destination.

This section analyzes the perception of tourists' destination image from the dimensions of intuition, positive emotion, and negative emotion. The specific dimensions are shown in Table 4.

Tourists' perception of the cognitive image of southern Xinjiang mainly focuses on natural tourism resources, special catering, climate environment, social environment, etc., and more of the praise of natural scenery and special food, which tends to be positive and emotional.

Through the extraction of emotional comment words and co-occurrence analysis, the positive and negative factors perceived by summer tourists are analyzed. Among the 30 emotional comment words extracted, high-frequency words such as “good,” “like,” “worthy,” “beautiful,” and “happy” reflect tourists' positive evaluation of the trip. “Enjoyment,” “stimulation,” “comfort,” and “comfortable” are the positive emotional expressions of tourists who escape from the usual environment to the tourist destination for vacation and leisure and enjoy the novel natural scenery and comfortable climate environment. However, due to weather factors, tourists are worried that they “cannot see what they want to see,” so they have emotional expressions of “regret,” “disappointment,” “missing,” and “gap.” In addition, due to the excessive passenger flow in the peak season, tourists also feel “dangerous,” “crowded,” and “tired.”

Tourism consumption is a typical hedonic consumption, experience consumption, the pursuit of feeling, fun, and pleasure, and tourism satisfaction mainly comes from experience, especially emotional experience. Rojas and Camarero believe that emotion is the determinant of satisfaction, and emotion has a moderating effect on satisfaction; Bosque believes that positive emotion and negative emotion are the antecedent variables of satisfaction, and loyalty is the dependent variable of satisfaction. Therefore, this study measures tourists' post-tour satisfaction evaluation from the two aspects of emotional tendency and behavioral willingness (i.e., loyalty).

To understand each tourist's sentiment evaluation of tourism, this section conducts sentiment analysis on text data based on document granularity and word granularity. First, the positive or negative sentiment words in each document are identified and scored through the sentiment dictionary, and then, the scores of all sentiment words in the document are aggregated and summed to obtain the final sentiment score. After the sentiment score statistics, the average sentiment score of the 500 travel notes is 46.73 points, of which the average positive (i.e., positive) sentiment score is 87.04 points, and the negative (i.e., negative) sentiment score is −40.31 points. Different emotional intensities are measured according to the sentiment score: positive affect (5, +∞), negative affect (−∞, −5), and neutral affect [−5, 5], where positive affect can be divided into high (25, +∞), moderate (15, 25], and moderate (5, 15); negative affect can be divided into high (−∞, −25), moderate [−25, −15), and moderate [−15, −5).

The statistical results in Figure 5 show that 91% of tourists have a positive emotional orientation towards the travel experience, of which 65% of tourists have the highest degree of positive emotion, 17% are moderate, and 18% are average. Only 1% of tourists have negative emotional inclinations, and all of them are highly negative, which shows that most tourists have positive and positive emotional inclinations towards the tourism experience in southern Xinjiang.

### 3.5. Behavioral Analysis-Based Tourism Development Strategies

Based on the two factors of geographic location and climate, the domestic primary market is the Bohai Rim Region with Beijing-Tianjin-Hebei as the core. This region has a developed economy, long high-temperature period in summer, and strong demand for summer vacation. The secondary market is the provinces and cities around scenario spots, and the travel distance in this area is short and suitable for short-term self-driving tourism products; the tertiary market is the Pearl River Delta region with Shanghai as the core, and travel in this area is long distance, developed economy, long high-temperature period, suitable for multi-destination in-depth tourism, and “airplane + other” combined transportation products; the fourth-level market is other domestic provinces and cities.

Relying on geographical advantages, “geo-tourism” is developed. Geo-tourism is developed, and characteristic border tourism products are created. Infrastructure construction is improved, tourism products are innovated and developed, the tourism industry chain is extended, and the “trade zone + tourism zone” construction is used to reduce travel barriers for tourists and promote the development of tourism.

Unique attractions are relied to develop “themed tourism.” Relying on the unique attractive elements of tourist destinations, we should develop characteristic-themed tourism products that meet the needs of different tourist groups: first is relying on the advantages of climate and environment and the second is to develop “food tourism” routes based on local catering characteristics. Finding, experiencing, and enjoying food have increasingly become an important tourist motivation.

Local cultural resources are relied to develop “cultural tourism”. Cultural tourism resources should be developed in the development of tourism resources, and cultural tourism forms such as historical exploration and folk customs should be developed using the unique local Korean culture, Kanto culture, national culture, and cultural resources and landscape resources. While satisfying the basic needs of tourists for sightseeing and taking pictures of beautiful scenery, it also develops tourism products with high participation and strong experience of tourists such as folk experience and adventure exploration, prolonging the length of tourists' stay, and satisfying tourists for summer vacation and vacation leisure purposes.

We should focus on making up for the shortcomings of infrastructure services, improving transportation service facilities, and improving the level of tourist reception services during peak seasons. First of all, in terms of tourism transportation, the accessibility of transportation is improved, especially the transportation accessibility outside the scenic spots, and the management of the order of the tourism transportation market is strengthened. Secondly, in terms of tourism commodities, there are many types of special products in tourist areas, but only blueberries and ginseng are mentioned in the travel notes. This shows that other special products cannot attract tourists' attention and desire to buy. The development and packaging of special products should be strengthened, as well as publicity. Finally, a connection mechanism for tourists in peak seasons is established to improve the quality and level of reception services for tourists in peak seasons, thereby reducing the safety risk of crowd congestion and the negative emotions of tourists.

Cooperation between cities and counties in tourist attractions in tourist areas is strengthened. Scenic spots and their management departments should strengthen the cooperation between core scenic spots and surrounding scattered scenic spots, establish a scenic spot cooperation mechanism, integrate scenic spots in tourist areas, extend outward from the core scenic spots tour routes, and implement a combined ticket or pass system in large tourist areas. The integrated development of regional tourism is promoted. Tourism cooperation outside tourist areas is strengthened. The tourism management department should strengthen the tourism linkage and cooperation with the tourism departments of other cities and jointly establish summer escape and border tourism routes or tourism strategies across the three northeastern provinces, to achieve a win-win situation for all parties.

Classified Internet marketing based on tourist segmentation: according to the degree of network involvement, tourists can be divided into high involvement and low involvement; according to the degree of experience, tourists can be divided into deep experience, moderate experience, and shallow experience; and according to age, tourists can be divided into teenagers, youth, middle-aged, and elderly; and according to the place of residence, tourists can be divided into the urban type and rural type. Different market segments have different motivations for online consumption, online consumption preferences, and online consumption perceptions and evaluations. Classification of online marketing strategies should be formulated according to the consumption habits and travel attitudes of different groups. For example, travel groups with high Internet involvement should cooperate with well-known and popular travel websites or online opinion leaders to increase the popularity of scenic spots in this area.

The factors that cause tourists' “dissatisfaction” are the concentrated congestion of tourists in peak season, which not only brings adverse effects on tourists' travel experience but also on the ecological environment of scenic spots. The best way to solve the problem of congestion is to accurately predict the flow of tourists, understand the spatial behavior of tourists, and implement tourist diversion.

There are still many deficiencies in this study, which need to be improved and further studied in future research. It is in terms of data: due to the limitation of data acquisition, 500 travel notes were obtained after screening, and the amount of data is not particularly large. In the future, more channels and methods will be explored to collect data, so that the reference value of the data will be more perfect; due to the influence of the personal privacy protection policy, personal information such as the age and knowledge level of the travel journal publisher cannot be accurately obtained, so the representativeness of the travel journal sample cannot be accurately measured; the travel journal includes text and image data. This article only studies the form of text data. The next step is to conduct research on the form of image data. In the future, data mining algorithms such as cluster analysis, topic identification and classification, and dependency modeling can be further studied and applied to in-depth study of tourist behavior patterns and mechanisms, as well as the establishment of an intelligent analysis system for tourist behavior based on UGC data.

## 4. Conclusions

By consulting, summarizing, and analyzing a large number of related literature studies on tourism consumer behavior, tourism big data, text data analysis, etc., this study constructs a thinking framework for the research of tourism consumption behavior based on UGC text data and conducts research on the basis of this thinking framework. We use train browser, NLPIR, and other software packages to crawl, preprocess, and travel sample data and use the word frequency analysis, co-occurrence analysis, content analysis, sentiment analysis, network analysis, and other methods to analyze the characteristics of tourists and decision-making. According to the behavior analysis, tourism management departments, and tourism enterprises, the reform and promotion of tourism marketing strategies and the improvement of tourism product and service quality were done. This study proposes the development strategy of southern Xinjiang summer vacation tourism in three aspects to improve the management mode of tourism destination. Finally, the conclusions of this study are as follows:

1. This study uses ten days as the unit to count the travel time and proposes to use ten days to months as the tourism cycle to develop tourism, refine product design, and adjust and allocate tourism resources.
2. Based on the “push-pull” theory, this study establishes a “push-pull resistance” tourism decision-making model. Through word frequency analysis, co-occurrence analysis, and content analysis, it is concluded that “escape” and “seek” are the internal driving forces that affect tourists' travel decisions. Among them, companionship and experience are the main travel motives. Tourism enterprises should develop and design in-depth and diversified experience products to create unforgettable travel experiences, thereby stimulating tourists' travel motivation: “climate suitability,” “attraction of scenic spots,” and “scenic spots.” “Uniqueness” is the pulling factor for tourists to choose the four destinations in southern Xinjiang. Scenic spots can use the pulling factor to create tourism IP and create “selling points” to attract tourists; in addition, the changeable weather and inconvenience of transportation have become obstacles for tourists to travel, so scenic spots should focus on making up for shortcomings and improving the quality of tourism services.
3. Through network analysis of scenic spots, it is found that there are three tourist routes preferred by tourists, namely short-distance travel and long-distance travel, and long-distance border travel. Tourism management departments and scenic spots should strengthen tourism cooperation between cities and scenic spots and develop theme tourism and diversified tourism routes such as geo-tourism and cultural tourism to achieve regional coordinated development.
4. Based on the “cognitive-emotional” model, this study describes the tourism image from two dimensions, cognitive image and emotional image. Generally, tourists present a positive perception state. In addition, this study measures tourist satisfaction from the analysis of emotional tendencies and future behavior intentions (i.e., loyalty, including willingness to revisit and recommendation). Emotional state but the revisit rate is not high, indicating that the tendency of post-tour memories and evaluations to be effectively transformed into re-consumption behavior is weak. Scenic spots or research communities can conduct in-depth research on the effective needs of tourists, and at the same time, the positive electronic word-of-mouth effect is used to adopt “tourism”. + new media,” “tourism + UGC,” and other marketing methods.
5. Based on the research on tourism consumer behavior based on UGC data, this study can help scenic spots and other tourism enterprises understand the consumption preferences of different tourism groups, optimize tourism routes, develop diversified tourism products, improve the quality of tourism services based on the characteristics and laws of tourists' behavior, and further cater to market segments.
6. This research provides a new idea for tourism scenic spots and tourism management departments to monitor tourists' behavior through big data analysis. A tourism big data analysis platform based on UGC data can be established to help relevant management entities to trace back the characteristics, changes in tourists' consumption behavior, and the impact on scenic spots. It can also help tourism websites to establish a personalized scenic spot recommendation system according to tourists' consumption preferences.

## Figures and Tables

**Figure 1:** 2015–2021 statistical statistics of online travel notes in southern Xinjiang.

**Figure 2:** Statistics of tourist travel days.

**Figure 3:** Statistics on per capita consumption of tourists.

**Figure 4:** Tourist attraction preference statistics based on word frequency and weight.

**Figure 5:** Statistical chart of emotional tendency analysis of travel notes.

**Table 1:** Statistical results of customer source distribution.

Distribution of tourists	Occur number	Frequency (%)
Northeast	160	32
North China	140	28
East China	102	20.4
Central South	58	11.6
Western South	12	2.4
Western North	8	1.6
Others	20	4
Total	500	100

**Table 2:** Word frequency statistics of tourist motivation.

	Weight	Frequency ofwords
*Pull factor*		
Kashgar Old Town	455.01	3259
Bayanbulak Grassland	279.5	1317
Tianshan Mysterious Grand Canyon	263	1438
Pamirs	185	730
Wensu Tomur Grand Canyon	124	340
Fragrant Concubine Garden	110	395
Xinjiang Robu Village Scenic Spot	108	400
Lop Nor	104	360
Kuqa Temple	90	344
Daolang Tribe	86	280
Kezier Thousand Buddha Caves	85	220
Loulan Ancient Town	83	89
Aksu Tianshan Sacred Wood Garden	69	230
Thousands of Miles of Grape Corridor	66	170
Bosten Lake	57	170
Taklimakan Desert	42	80
Kuqa Old Town	34	130
Muztagh	34	40
Karakul Lake	30	90
Tarim Populus Euphratica Park	23	200
Datongxiang Apricot Flower	22	180
Karakoram Highway	20	140
Taxkorgan Baisha Lake	18	60
Kashgar Ferris Wheel	18	130
Edgebrook Swan Lake	17	150
Muji Crater	14	90
Niya Ruins	12	130
Taxkorgan Town	10	100
Iron Gate	7	70
Bayanbulak Reserve	6	40

*Thrust factor*		
Friends	127	300
Children	107	320
Experience	101	220
Summer	85	270
Hot summer	40	120
High temperature	35	50
Climb mountains	33	210
Fascinated	27	60
Escape	24	50
Entertainment	23	70
Go away	22	70
Visiting	20	130
Feel	19	140
Appreciate	18	140
Relax	18	60
Parents	18	110
Seek	16	50
Enjoy	16	130
Vacation	15	320
Stimulate	14	100
Freedom	9	150

*Resistance factor*		
Weather	165	560
Traffic	95	290
Can't see the most wanted scenery	33	80
Bad weather	16	10
Changeable weather	13	20
Pity	10	120
Inconvenient traffic	4	22
Black car	4	15

**Table 3:** Keyword extraction and analysis of tourism information channels.

Keywords	Weight	Frequency of words
Raiders	104	250
Travel APP	58	80
Ctrip	51	90
Where to	43	90
Public comment	27	35
Online/Web	22	370
Travel notes	20	500
Baidu map	19	22
Hornet's nest	11	25
Website/official website	15	40
Baidu	7	30
Taobao	5	20

**Table 4:** Analysis of intuition dimension, positive affective dimension, and negative affective dimension.

Tourism perception	Dimension	Keyword weight and word frequency	Co-occurrence word pair and word frequency
	Cognitive dimension (total word frequency 2488)	Beautiful, delicious, beautiful, spectacular, lung washing, clean, natural, beautiful, cool, mysterious, enthusiasm, blue sky and white clouds, open, beautiful, magical, full view of Tianchi, beautiful, fairyland, holy, spectacle, beautiful, fresh air, natural oxygen bar	Korean cuisine/northeastern cuisine—delicious (72); northeasterner/service staff/staff—enthusiastic (50); Grand Canyon—spectacular (45); mountain top—holy (46); environment—quiet (25)
	Positive (total word frequency 2806)	Feeling, good, like, worthy, lucky, enjoy, hope, comfortable, exciting, beautiful, comfortable, happy, anticipation, shock, comfort, excitement, gratitude, surprise	Worth—recommended/experience/share/see (134); taste/taste—good (68); scenery/environment—good (50); air/environment—comfort (26); nature/travel/food (26); weather—nice (9)
	Negative (total word frequency 1087)	average, bad, regret, worry, can't see the scenery, missed, disappointment, disappointment, regret, tired, dangerous, crowded	Weather/luck/road condition—bad (44); no view/stay—regret (29); worry—no view/weather/time (27); scenic/crowd—crowded (24)

## Data Availability

The experimental data used to support the findings of this study are available from the corresponding author upon request.
